# Melatonin improves mitochondrial biogenesis through the AMPK/PGC1α pathway to attenuate ischemia/reperfusion-induced myocardial damage

**DOI:** 10.18632/aging.103078

**Published:** 2020-04-19

**Authors:** Xueyan Qi, Jin Wang

**Affiliations:** 1 Department of Cardiology, Tianjin First Central Hospital, Tianjing 300192, China; 2 Department of Cardiology, the First Medical Center, Chinese PLA General Hospital, Beijing 100853, China

**Keywords:** melatonin, mitochondrial biogenesis, mitochondrial dysfunction, ischemia-reperfusion injury

## Abstract

Cardiac ischemia/reperfusion injury is associated with reduced mitochondrial turnover and regeneration. There is currently no effective approach to stimulate mitochondrial biogenesis in the reperfused myocardium. In this study, we investigated whether melatonin could increase mitochondrial biogenesis and thus promote mitochondrial homeostasis in cardiomyocytes. Cardiomyocytes were subjected to hypoxia/reoxygenation (H/R) injury with or without melatonin treatment, and various mitochondrial functions were measured. H/R injury repressed mitochondrial biogenesis in cardiomyocytes, whereas melatonin treatment restored mitochondrial biogenesis through the 5’ adenosine monophosphate-activated protein kinase (AMPK)/peroxisome proliferator-activated receptor-gamma coactivator 1 alpha (PGC1α) pathway. Melatonin enhanced mitochondrial metabolism, inhibited mitochondrial oxidative stress, induced mitochondrial fusion and prevented mitochondrial apoptosis in cardiomyocytes subjected to H/R injury. The melatonin-induced improvement in mitochondrial biogenesis was associated with increased cardiomyocyte survival during H/R injury. On the other hand, silencing of *PGC1α* attenuated the protective effects of melatonin on cardiomyocyte viability, thereby impairing mitochondrial bioenergetics, disrupting the mitochondrial morphology, and activating mitochondrial apoptosis. Thus, H/R injury suppressed mitochondrial biogenesis, while melatonin activated the AMPK/PGC1α pathway and restored mitochondrial biogenesis, ultimately protecting the reperfused heart.

## INTRODUCTION

Myocardial ischemia/reperfusion (I/R) injury occurs at the stage of reperfusion due to reactive oxygen species (ROS) overproduction, calcium overload, the inflammatory response and microvascular damage [1, 2]. Mitochondria contribute to myocardial I/R injury by inducing various pathological processes [3–8]. First, most ROS are generated and released by mitochondria when electron transport chain activity is reduced. Second, mitochondria serve as calcium pumps in cardiomyocytes, so they can contribute to intracellular calcium overload when the mitochondrial calcium uniporter is dysregulated. Third, mitochondria-induced oxidative stress and cardiomyocyte death initiate an inflammatory response to repair the damaged myocardium. Fourth, although the content of mitochondria in endothelial cells is relatively low, mitochondrial morphologic disorder has been observed in cardiac microvascular injury following I/R injury. Therefore, several studies have identified mitochondria as the primary targets of strategies to prevent cardiac I/R damage.

Mitochondria are renewable organelles. Damaged mitochondrial fragments can be metabolized by mitophagy and then regenerated through mitochondrial biogenesis [9–11]. Mitophagy determines the degradation rate of old mitochondria, whereas mitochondrial biogenesis sustains mitochondrial population turnover [12–14]. Defective mitophagy has been observed in cardiac I/R injury, and is associated with mitochondrial dysfunction in cardiomyocytes and cardiac microvascular endothelial cells [15, 16]. Similarly, mitochondrial biogenesis was found to be inhibited in a mouse model of cardiac I/R injury; thus, improving mitochondrial biogenesis is considered to be a promising method of alleviating cardiac I/R injury [17, 18]. However, there is not yet an effective drug to promote mitochondrial biogenesis in the heart.

Melatonin, a biological rhythm-related hormone, significantly protects the heart against cardiac I/R injury [19, 20]. The cardioprotective mechanisms of melatonin include the protection of mitochondria, the suppression of inflammation and the inhibition of oxidative stress [21–25]. Mitochondria seem to be the first targets of melatonin treatment [26–28]. Melatonin can normalize mitochondrial oxidative stress, thus stabilizing the mitochondrial membrane potential and promoting adenosine triphosphate (ATP) synthesis. In addition, melatonin regulates mitochondrial morphological alterations such as fission and fusion in the heart during I/R injury. Melatonin also improves mitophagy by inducing optic atrophy 1 (OPA1), FUN14 domain containing 1 and Parkin [7, 21, 29, 30]. Thus, melatonin promotes mitochondrial homeostasis.

Although melatonin has been reported to accelerate mitochondrial biogenesis in early porcine embryos [31], differentiating rat dental papilla cells [32] and Alzheimer’s disease patients [33], its involvement in mitochondrial biogenesis in the setting of cardiac I/R injury has not been investigated. In the present study, we performed cellular experiments to explore the influence of melatonin on mitochondrial biogenesis in cardiac I/R injury.

## RESULTS

### Mitochondrial biogenesis impaired by hypoxia/reoxygenation (H/R) injury could be improved by melatonin

To assess the alterations in mitochondrial biogenesis following H/R injury, we subjected cardiomyocytes to six-hour hypoxia and six-hour reoxygenation. Then, we performed quantitative real-time PCR (qRT-PCR) and immunoblotting to analyze parameters associated with mitochondrial biogenesis. As shown in Figure 1A–1C, the mRNA levels of peroxisome proliferator-activated receptor-gamma coactivator 1 alpha (*PGC1α*), transcription factor A mitochondrial (*Tfam*) and nuclear factor erythroid 2-related factor 2 (*Nrf2*) were significantly lower in the H/R injury group than in the control group. Melatonin treatment dose-dependently increased *PGC1α*, *Tfam* and *Nrf2* levels in H/R-injured cells (Figure 1A–1C). We also evaluated the mRNA levels of *Sirt3*, a novel biomarker of mitochondrial biogenesis. *Sirt3* levels in cardiomyocytes were notably reduced after H/R injury, but were restored following melatonin treatment (Figure 1D). Due to the reduced transcription of *PGC1α*, *Tfam* and *Nrf2*, the protein levels of translocase of inner mitochondrial membrane 23 (Tim23) and translocase of outer mitochondrial membrane 20 (Tom20) were also reduced in cardiomyocytes subjected to H/R injury, suggesting that the mitochondrial mass had decreased (Figure 1E and 1F). Melatonin treatment restored the expression of Tim23 and Tom20 (Figure 1E and 1F). These data indicate that melatonin can normalize mitochondrial biogenesis during H/R injury.

**Figure 1:** **Melatonin treatment restores mitochondrial biogenesis in H/R-treated cardiomyocytes.** Cardiomyocytes were subjected to H/R injury, with or without previous melatonin treatment to protect the cardiomyocytes. (**A**–**D**) qPCR assays were used to evaluate the transcription of *PGC1α*, *Tfam*, *Nrf2* and *Sirt3*. (**E**, **F**) Western blots were used to evaluate the alterations in the mitochondria-related proteins Tom20 and Tim23. *p<0.05.

### Melatonin promotes mitochondrial biogenesis by inducing the 5’ adenosine monophosphate-activated protein kinase (AMPK) pathway

To determine the molecular basis for the above findings, we analyzed the expression of upstream regulators of PGC1α. Since the AMPK signaling pathway post-transcriptionally modifies PGC1α, we performed an enzyme-linked immunosorbent assay (ELISA) to detect AMPK activity in cardiomyocytes in response to H/R injury. As shown in Figure 2A, AMPK activity was significantly lower in the H/R injury group than in the control group; however, melatonin treatment restored AMPK activity. An immunofluorescence assay confirmed that the expression of phosphorylated (p)-AMPK was reduced in cardiomyocytes exposed to H/R injury, but was restored by melatonin treatment (Figure 2B and 2C).

**Figure 2:** **Melatonin activates the AMPK pathway to induce mitochondrial biogenesis.** Cardiomyocytes were subjected to H/R injury, with or without previous melatonin treatment to protect the cardiomyocytes. (**A**) An ELISA was used to evaluate AMPK activity. (**B**, **C**) An immunofluorescence assay was used to evaluate the expression of p-AMPK. (**D**, **E**) qPCR was used to evaluate the transcription of *Tfam* and *Nrf2*. CC was used to inhibit the activity of AMPK. *p<0.05.

To determine whether AMPK was required for melatonin-induced mitochondrial biogenesis, we used compound c (CC) to inhibit AMPK activity in cardiomyocytes. Blocking the AMPK pathway suppressed the melatonin-induced increases in *Tfam* and *Nrf2* mRNA levels (Figure 2D and 2E). CC supplementation also abolished the melatonin-induced increase in the mitochondrial mass (Figure 2D and 2E). Thus, AMPK was required for melatonin-induced mitochondrial biogenesis in H/R-treated cardiomyocytes.

### Silencing of *PGC1α* abolishes the protective effects of melatonin on mitochondrial bioenergetics

Next, we assessed the effects of mitochondrial biogenesis on mitochondrial function in cardiomyocytes damaged by H/R injury. Since our earlier findings indicated that melatonin induced *PGC1α*, we used small interfering RNA (siRNA) to silence *PGC1α* in cardiomyocytes. We found that mitochondrial ATP production in cardiomyocytes was reduced by H/R treatment and restored by melatonin treatment; however, the effects of melatonin were nullified when *PGC1α* was knocked down (Figure 3A). Given that ATP levels were reduced upon H/R injury, we then measured mitochondrial ROS production in cardiomyocytes. As shown in Figure 3B and 3C, mitochondrial ROS fluorescence was greater in the H/R group than in the control group; however, melatonin attenuated mitochondrial ROS production. Notably, when melatonin-treated H/R-injured cardiomyocytes were transfected with siRNA against *PGC1α*, mitochondrial ROS fluorescence increased again (Figure 3B and 3C). The mitochondrial membrane potential in cardiomyocytes was also reduced in response to H/R injury (Figure 3D and 3E). Melatonin treatment stabilized the mitochondrial membrane potential, but not in *PGC1α*-silenced cells (Figure 3D and 3E). These data indicate that melatonin enhanced mitochondrial bioenergetics and suppressed oxidative stress by inducing *PGC1α*.

**Figure 3:** **Melatonin preserves mitochondrial function in H/R-treated cardiomyocytes by inducing the AMPK/PGC1α pathway.** Cardiomyocytes were subjected to H/R injury, with or without previous melatonin treatment to protect the cardiomyocytes. The cardiomyocytes were transfected with siRNA to knock down *PGC1α*. (**A**) An ELISA was used to assess ATP production. (**B**, **C**) An immunofluorescence assay was used to measure mitochondrial ROS in cardiomyocytes. (**D**, **E**) An immunofluorescence assay was used to measure the mitochondrial membrane potential. *p<0.05.

**PGC1α-induced mitochondrial biogenesis also alters the mitochondrial morphology**

In addition to monitoring mitochondrial function, we assessed the mitochondrial morphology in cardiomyocytes. As shown in Figure 4A and 4B, H/R injury induced mitochondrial fragmentation, suggesting that H/R injury either increased mitochondrial fission or reduced mitochondrial fusion. The average length of the mitochondrial mass was lower in the H/R group than in the control group (Figure 4A and 4B). Melatonin treatment inhibited the formation of fragmented mitochondria and thus sustained the mitochondrial length; however, this effect depended on the expression of *PGC1α* (Figure 4A and 4B). At the molecular level, H/R injury significantly repressed the transcription of mitofusin 2 (*Mfn2*) and *Opa1*, whereas melatonin upregulated these genes (Figure 4C and 4D). Loss of *PGC1α* abolished the melatonin-induced upregulation of *Mfn2* and *Opa1*. These data indicate that mitochondrial biogenesis restored mitochondrial fusion in H/R-treated cardiomyocytes.

**Figure 4:** **Melatonin alters the mitochondrial morphology in cardiomyocytes by inducing the AMPK/PGC1α pathway.** Cardiomyocytes were subjected to H/R injury, with or without previous melatonin treatment to protect the cardiomyocytes. The cardiomyocytes were transfected with siRNA to knock down *PGC1α*. (**A**, **B**) An immunofluorescence assay was used to assess the mitochondrial morphology. (**C**, **D**) A qPCR assay was used to evaluate the transcription of *Opa1* and *Mfn2*. (**E**, **F**) An mt-kemia assay was used to evaluate mitophagy activity. *p<0.05.

Next, we used the mt-kemia assay to observe the level of mitophagy in H/R-treated cardiomyocytes. As shown in Figure 4E and 4F, mitophagy was downregulated in the H/R injury group compared with the control group, as evidenced by the reduced number of acidic mitochondria in cardiomyocytes. Melatonin restored mitophagy activity, but the loss of *PGC1α* prevented the melatonin-induced upregulation of mitophagy in cardiomyocytes (Figure 4E and 4F). These results indicate that melatonin normalized the mitochondrial morphology in H/R-treated cardiomyocytes.

### Melatonin requires PGC1α-induced mitochondrial biogenesis to inhibit mitochondrial apoptosis in H/R-treated cardiomyocytes

Damaged mitochondria are associated with cardiomyocyte death. Therefore, we evaluated the anti-apoptotic effects of mitochondrial biogenesis. Caspase-9 activity increased rapidly in response to H/R injury, and melatonin prevented this alteration (Figure 5A). However, when *PGC1α* was silenced, caspase-9 was re-activated in melatonin-treated cardiomyocytes (Figure 5A). The opening rate of the mitochondrial permeability transition pore (mPTP) also increased in response to H/R injury. Melatonin treatment reduced the mPTP opening rate in a manner dependent on *PGC1α* expression (Figure 5B).

**Figure 5:** **Melatonin-induced mitochondrial biogenesis promotes cardiomyocyte survival.** Cardiomyocytes were subjected to H/R injury, with or without previous melatonin treatment to protect the cardiomyocytes. The cardiomyocytes were transfected with siRNA to knock down *PGC1α*. (**A**) An ELISA was used to assess caspase-9 activity. (**B**) The mPTP opening rate was determined in cardiomyocytes. (**C**, **D**) TUNEL staining for apoptotic cells in cardiomyocytes. (**E**, **F**) An immunofluorescence assay was used to measure the expression of myosin. *p<0.05.

Due to the increased mPTP opening rate and elevated caspase-9 activity, the number of terminal deoxynucleotidyl transferase dUTP nick end labeling (TUNEL)-positive cells was greater in the H/R group than in the control group (Figure 5C and 5D). Fewer apoptotic cells were found in the melatonin group, but the loss of *PGC1α* abolished the inhibitory effect of melatonin on mitochondrial apoptosis. More importantly, H/R injury significantly reduced the fluorescence intensity of myosin (Figure 5E and 5F), indicating that the cardiomyocyte cytoskeleton had been degraded. Melatonin treatment increased the expression of myosin by upregulating *PGC1α*, confirming that melatonin exerted anti-apoptotic effects on cardiomyocytes during H/R injury. These results indicate that melatonin inhibited mitochondrial apoptosis in H/R-treated cardiomyocytes by stimulating PGC1α-induced mitochondrial biogenesis.

## DISCUSSION

In order to pump blood, cardiomyocytes require mitochondria; therefore, mitochondrial homeostasis is vital for cardiomyocyte function. Many studies have demonstrated that enhancing mitochondrial activity is a promising strategy to improve cardiomyocyte viability and cardiac function during myocardial I/R injury. Cardiac I/R injury has been attributed to three molecular mechanisms: cardiomyocyte death, inflammation and oxidative stress [34–38]. However, defective energy metabolism and microvascular damage have also been noted in the reperfused heart [39–41].

Mitochondria seem to be involved in every aspect of the various physiological and pathological events during the development of cardiac I/R injury. For example, mitochondria can induce cardiomyocyte death by releasing pro-apoptotic proteins and activating the endogenous apoptotic pathway. Oxidative stress is primarily caused by ROS overload, and mitochondria are the main producers of ROS through impaired oxidative phosphorylation [42]. Mitochondrial damage-induced oxidative stress also promotes cardiomyocyte death by inducing membrane oxidation and protein post-transcriptional modifications. The inflammatory response may be secondary to cardiomyocyte death and oxidative stress, because the inflammatory response is triggered by inflammatory cell accumulation, which results from cardiomyocyte apoptosis [43–45]. Therefore, mitochondrial homeostasis is linked to the extent of cardiac I/R injury.

Mitochondrial homeostasis is maintained through structural and functional alterations. Mitochondrial morphological adaptions (also known as mitochondrial dynamics) include mitochondrial fission, fusion and mitophagy [46–49], and have been carefully discussed in several articles [50–52]. In this study, we explored the contribution of mitochondrial biogenesis to mitochondrial homeostasis. Mitochondrial biogenesis regenerates mitochondria and ultimately increases the mitochondrial mass, as evidenced by increased levels of mitochondrial DNA and mitochondria-related proteins [53, 54]. Mitochondrial biogenesis rapidly augments the mitochondrial population in a short time, which is necessary for cell metabolism under stress. Although several studies have described the alterations in mitochondrial biogenesis in the setting of cardiac I/R injury [55–57], the protective mechanism of mitochondrial biogenesis has not been fully elucidated. Herein, we found that mitochondrial biogenesis was inhibited in cardiomyocytes subjected to H/R injury. Consequently, mitochondrial bioenergetics were impaired, the mitochondrial morphology was disrupted and mitochondrial function was reduced. Improving mitochondrial biogenesis elevated cardiomyocyte ATP production, prevented mitochondrial fragmentation, enhanced mitochondrial function, stimulated mitophagy and inhibited mitochondrial apoptosis. Therefore, mitochondrial biogenesis may be a critical determinant of mitochondrial structure, function and homeostasis.

Melatonin is an effective drug for the treatment of cardiac I/R injury. Cytoplasmic melatonin can accumulate in the mitochondria and enhance mitochondrial redox balance and bioenergetics. Although melatonin is thought to sustain mitochondrial function through its anti-oxidative actions, melatonin also controls mitochondrial fission, fusion, mitophagy, apoptosis, necroptosis and calcium balance during cardiac I/R injury. In this study, we observed that melatonin stimulated mitochondrial biogenesis. Melatonin activated the AMPK pathway, which thus upregulated *PGC1α*, *Tfam*, *Nrf2* and *Sirt3*. Tfam, Nrf2 and Sirt3 have been reported to increase mitochondrial DNA levels and oxidative phosphorylation-related protein translation. Melatonin treatment also increased the mitochondrial mass and improved mitochondrial function. Thus, we have provided a method of restoring mitochondrial biogenesis in the reperfused heart.

There are several limitations to our experiments. First, we did not obtain animal data to support the function of mitochondrial biogenesis in the reperfused heart. Second, we only tested the effects of one concentration of melatonin on mitochondrial biogenesis. Nevertheless, our results indicated that melatonin improved mitochondrial biogenesis and promoted the transmission of protective signals for mitochondria in H/R-treated cardiomyocytes.

## MATERIALS AND METHODS

### Cell isolation, culture, treatment and transfection

Primary cultures of neonatal mouse ventricular cardiomyocytes were prepared from the ventricles of three- to five-day-old mice as described previously [58]. Cardiomyocytes were plated on type I collagen-coated cover glasses or culture plates, and were incubated with Dulbecco’s modified Eagle’s medium supplemented with bovine serum albumin or palmitate-bovine serum albumin. Cardiomyocytes were also transfected with siRNA against *PGC1α*. After 12 hours of transfection, the cardiomyocytes were incubated in Dulbecco’s modified Eagle’s medium with or without palmitate, as described above. H/R injury was induced through six-hour hypoxia and six-hour reoxygenation, as previously described. Melatonin (5 μM) was used 12 hours prior to H/R treatment. CC (10 μM, Selleck Chemicals, Houston, TX, USA) was added to the medium for two hours to prevent AMPK activation [59].

### Mitochondrial function

Mitochondrial function was evaluated with a JC-1 Mitochondrial Membrane Potential kit (Cayman Chemical) according to the manufacturer’s instructions. An ELISA was performed, and the signal was detected on a plate reader (EnSpire® Multimode Plate Reader, Perkin Elmer).

The extracellular oxygen consumption rate was evaluated with a fluorescence-based oxygen consumption rate assay kit (Abcam) according to the manufacturer’s instructions [60]. Briefly, cells were treated with 20 μM octyl-α-ketoglutarate or 10 μM AA6. Dimethyl sulfoxide was used as a solvent. The fluorescent signal was detected every minute for one hour on a multi-well plate reader (EnSpire® Multimode Plate Reader) set at 37 °C, excitation/emission=380/650 nm. Signals were normalized to the total DNA content, which was assessed with DRAQ5 (1:1000, Biostatus) [61].

### Immunofluorescence and confocal microscopy

Confocal analysis was performed as reported previously. Paraffin-embedded and cryosectioned samples were prepared according to standard histological procedures [62]. Mitochondria were visualized with MitoTracker Red CMXRos (1:2000, Thermo Scientific) and JC-1 (5 μM, AdipoGen). The samples were analyzed on a Leica TCS SP8 confocal microscope [63].

### Cell counting kit-8 (CCK-8) assay

A CCK-8 assay was used to assess cell viability [64]. Briefly, adherent cells were detached with trypsin, seeded in 96-well plates at 5×10^3^ cells/well, and allowed to attach to the bottom of the plate for 24 hours at 37 °C. The cells were then subjected to H/R injury with or without melatonin. Lastly, the cell viability was measured at 450 nm using CCK-8 [65].

### Western blotting

Western blotting was performed as described previously. Briefly, samples were lysed in complete radioimmunoprecipitation assay buffer (10 mM Tris-HCl pH 7.4, 150 mM NaCl, 1% NP40, 0.1% sodium dodecyl sulfate, 1 mM phenylmethylsulfonyl fluoride and 1x protease inhibitor cocktail [Roche]) and homogenized with a Sonic Dismembrator 100 (Fisher Scientific) [66]. The protein concentration of the sample homogenate was measured with a Bio-Rad Protein Assay, and equal amounts of soluble proteins were separated on 10% polyacrylamide gels, transferred onto nitrocellulose membranes and subjected to routine Western blot analysis [67].

### TUNEL staining

The paraffin-embedded sections obtained from the experiment above were dewaxed with fresh xylene (twice, for 10 min each) and dehydrated using a serial alcohol gradient [68]. Then, the tissue slides were treated with 20 μg/mL DNase-free protease K, incubated at 20-37 °C for 15-30 min, and washed three times with phosphate-buffered saline [69]. Then, 50 μL of TUNEL solution was added to the tissue slides, and the slides were incubated at 37 °C for 60 min in the dark. After being washed three times with phosphate-buffered saline, the slides were treated with an anti-fluorescence quenching agent and observed via fluorescence microscopy at an excitation wavelength of 450-500 nm and an emission wavelength of 515-565 nm [70].

### qRT-PCR analysis

An RNAiso Plus Purification Kit (TaKaRa Biotechnology Co., Ltd, 9108) was used to extract total RNA from the cardiomyocytes. The RNA concentration was evaluated based on the optical density of the sample at 260 nm, and the RNA integrity was assessed through 2% agarose gel electrophoresis. The RNA was reverse-transcribed into cDNA using a PrimeScript™ RT Reagent Kit with gDNA Eraser (TaKaRa Biotechnology Co., Ltd, RR047A) [71, 72]. Real-time PCR was performed on a LightCycler machine (Roche) with a commercial SYBR Green reaction reagent (TaKaRa Biotechnology Co., Ltd, RR820A). *GAPDH* was used as an internal control. The cDNA was denatured for 30 s at 95 °C, followed by 40 cycles of 5 s at 95°C [73].

### Statistical analysis

Statistical analyses were performed with GraphPad Prism. The sample sizes (n) are reported in the corresponding figure legends. The present study was exploratory and primarily mechanistic. For all analyses, the observer was blind to the identity of the samples. The variables were analyzed using non-parametric Student’s t-tests or analysis of variance (one-way or two-way). A value of p<0.05 was deemed statistically significant. Results are shown as the mean ± standard error.
